# Facial Features Detection System To Identify Children With Autism Spectrum Disorder: Deep Learning Models

**DOI:** 10.1155/2022/3941049

**Published:** 2022-04-04

**Authors:** Zeyad A. T. Ahmed, Theyazn H. H. Aldhyani, Mukti E. Jadhav, Mohammed Y. Alzahrani, Mohammad Eid Alzahrani, Maha M. Althobaiti, Fawaz Alassery, Ahmed Alshaflut, Nouf Matar Alzahrani, Ali Mansour Al-madani

**Affiliations:** ^1^Department of Computer Science, Dr. Babasaheb Ambedkar Marathwada University, India; ^2^Applied College in Abqaiq, King Faisal University, P.O. Box 400, Al-Ahsa 31982, Saudi Arabia; ^3^Shri Shivaji Science & Arts College, Chikhli Dist. Buldana, India; ^4^Department of Computer Sciences and Information Technology, Albaha University, Albaha, P.O. Box 1988, Saudi Arabia; ^5^Department of Engineering and Computer Science, Al Baha University, Albaha, P.O. Box 1988, Saudi Arabia; ^6^Department of Computer Science, College of Computing and Information technology, Taif University, P.O.Box 11099, Taif 21944, Saudi Arabia; ^7^Department of Computer Engineering, College of Computers and Information Technology, Taif University, P.O. Box 11099, Taif 21944, Saudi Arabia; ^8^College of Computer Science and Information Technology, Albaha University, Albaha, P.O. Box 1988, Saudi Arabia

## Abstract

Autism spectrum disorder (ASD) is a neurodevelopmental disorder associated with brain development that subsequently affects the physical appearance of the face. Autistic children have different patterns of facial features, which set them distinctively apart from typically developed (TD) children. This study is aimed at helping families and psychiatrists diagnose autism using an easy technique, viz., a deep learning-based web application for detecting autism based on experimentally tested facial features using a convolutional neural network with transfer learning and a flask framework. MobileNet, Xception, and InceptionV3 were the pretrained models used for classification. The facial images were taken from a publicly available dataset on Kaggle, which consists of 3,014 facial images of a heterogeneous group of children, i.e., 1,507 autistic children and 1,507 nonautistic children. Given the accuracy of the classification results for the validation data, MobileNet reached 95% accuracy, Xception achieved 94%, and InceptionV3 attained 0.89%.

## 1. Introduction

Developmental disorders are chronic disabilities that have a critical impact on many people's daily performance. The number of people with autism is increasing around the world, which leads families to have increased anxiety about their children and requires an examination to ensure the health of their children if they are autistic. An autistic patient needs special care in order to develop perceptual skills to communicate with their family and society. When an autistic patient is diagnosed at an early stage, the results of behavioral therapy will be more effective. Scientists at the University of Missouri, who studied the diagnosis of children using facial features [1], found that autistic children share common distinctive facial feature compared to children without autism (nonautistic children). Those features are an unusually broad upper face, including wide-set eyes, and a shorter middle region of the face, including the cheeks and nose.  Figure 1 shows the differences in facial features between children with autism in the first row and nonautistic children in the second row. Those images were taken from the Kaggle database, which was used in this study.

Recognizing developmental disorders from the image of a face is a challenge in the field of computer vision. Autism spectrum disorder (ASD) is a neurological problem that affects the child's brain from an early age. The autistic children suffer from difficulties in speech and social interaction, including difficulty establishing the correct visual focus of attention [1]. Those problems can be detected after 36 months. The challenge is how to provide an accurate diagnosis. Artificial intelligence is characterized by speed of decision-making and a reduction in the time required to make a diagnostic compared to traditional methods of diagnoses to detect autism in the early stage of life. The process of making an autism diagnosis is manual, and it is based on psychologists observing the behavior of a child for a long time. Sometimes this task takes more than two sessions. The development of technology has enabled the development of screening and diagnostic mechanisms to diagnose autism. The development of artificial intelligence has led to its increased use in the field of health and medical care, and researchers are very engaged in developing methods to diagnose ASD and detect autism at an early age using different technologies [2], such as brain MRI, eye tracking, electroencephalogram (EEG) signals, and eye contact [3]. A few researchers have used facial features to detect autism. Examples of differences in facial features are presented in Figure 1.

Currently, artificial intelligence has played the significant role for developing computer-aided diagnosis of autism [4–11] and moreover developing interactive system to assistance in the reintegration and treatment of autistic patients [12–14]. A number of researchers have applied machine learning algorithms for classification autism, such as schizophrenia [15–18], dementia, depression [19], autism [20–24], ADHD [25], and Alzheimer's [26] by using MRI.

The main objective of this study was to develop a deep learning-based web application using a convolutional neural network with transfer learning to identify autistic children using facial features. This application was designed to help families and psychiatrists to diagnose autism easily and efficiently. The current study applied one of the most popular deep learning algorithms, called CNN, to the Kaggle dataset. The dataset consists of images of faces divided into classes: autistic and nonautistic children. The face of a human being has many features that can be used to recognize identity, behavior, emotion, age, and gender. The researchers of this study used facial features to develop a deep learning model to classify autistic and nonautistic children based on their faces.

The diagnosis of Autism can be done using different techniques, such as brain MRI, eye-tracking, EEG, and eye contact [3].  Figure 2 shows autism detection techniques. This section reviews some previous studies that used facial features to detect autism. The methodologies are based on three perspectives. First, studies based on the facial features from the image of a face; Praveena and Lakshmi [2], Yang [27], and Beary et al. [28] developed deep learning models using online images of faces of autistic children and nonautistic children. Grossard et al. [29] found a different pattern distributed in the eyes and mouth in the image data of two groups: ASD and TD children. [27] used a pretraining model, which achieved 94% accuracy on validation data. Grossard et al. [29] achieved 90% accuracy with his classifier model. Beary et al. [28] used the VGG19 pretraining model, which achieved 0.84% accuracy on validation data. Haque and Valles [30] implemented a ResNet50 pretraining model on a small dataset, which consisted of 19 TD and 20 ASD children and achieved 89.2% accuracy. Some different techniques that have been used to detect the autism are presented in Figure 2.

## 2. Materials and Methods

Children with autism have different patterns of facial features, and the distance between facial landmarks and the width of landmarks is different compared to TD children.  Figure 3 displays the framework of the proposed system to identify autism from different human faces. Deep learning techniques are used to extract these subtle facial features and classify children into autistic and nonautistic groups. This study is based on CNN, which can learn the essential shapes in the first layers and improve the image's learning features in the deeper layers, to access accurate image classification. In other words, the feature extraction is done automatically through the CNN layers [31]. The advantages of the pretraining model are reducing the time needed to build and train the model from scratch. It is also good for achieving high accuracy with a small dataset, such as the one used in this study.

### 2.1. Dataset

This paper used a publicly available dataset from Kaggle [32]. This dataset consists of 3,014 images of faces, 1,507 of autistic and 1,507 of nonautistic children, as described in Figure 4. The images of the faces of autistic children were collected from online sources related to autism disorder, and the images of the faces of nonautistic children were randomly collected from the Internet.  Figure 5 shows numbers of examples used to evaluate the proposed system.

### 2.2. Preprocessing

The preprocessing of the dataset was done by the dataset creator to remove duplicated images and crop the images to show only the face, as shown in Figure 2. The dataset was then divided into three categories: 2,654 for training, 280 for validation, and 80 for testing. After obtaining the data, Keras preprocessing Image Data Generator normalized the dataset by rescaling the parameters, which scaled all the images in the dataset based on pixel values from [0, 255] to [0,1]. The reason for normalizing was to make the dataset ready for training using the CNN model.

### 2.3. Convolutional Neural Network Models

This section gives an overview of convolutional neural network architecture and the CNN pretraining models.

The convolutional layer is an important part of the CNN model that is used for feature extraction. The first convolutional layer learns basic features: edges and lines. The next layer extracts the features of squares and circles. More complex features are extracted in the following layers, including the face, eyes, and nose. The basic components of the CNN model are the input layer, convolutional layer, activation function, pooling layer, fully connected layer, and output prediction.

#### 2.3.1. Pooling Layer

When the CNN has a number of the hidden layers, that increases the depth of the output layer, so parameters of the CNN are large, requiring optimization of the mathematical operations space complexity and time of learning process. The pooling layer reduces the number of the parameters in the output from the convolution layer, using a summary statistical function. There are two types of pooling layers: Max-pooling and Average-pooling. Max-pooling takes the maximum values in each window in stride, as shown in Figure 6. Average-pooling calculates the mean value of each window in stride. In this case, the input to the next layer reduces the feature map, as shown in Figure 5.

#### 2.3.2. Fully Connected Layer

The fully connected layer receives the output from the convolutional layer and pooling layer, which have all the features, and puts them in a long tube.  Figure 7 shows the fully connected layer.

#### 2.3.3. Activation Function

The activation function classifies the output. The SoftMax activation function classifies the output when the number of classes is two or more. In this study, there are two classes: ASD and TD. The sigmoid activation function can be used with binary classification problems. The activation function is calculated using formula (1). This formula is called the slope and intercept of a line.  Figure 8 shows a diagram of the activation function.

(1) $$\begin{array}{c} y=x1*w1+x2*w2+b, \end{array}$$

where *x* is training data and *w* is weighetd of neural network. For output prediction, the results of the CNN model, after training, predicate the input image (ASD or TD) in our study.

### 2.4. Pretraining Models

This study implemented different CNN pretraining models for autism detection using images of faces. Then, the results were compared to select the best performing model.

Transfer learning uses the architecture and the weight of the model, which is trained on a large database and achieves high accuracy; then, it is used to solve a similar problem. The pretrained model sometimes takes a long time; it can take weeks to train using a large dataset and high configuration computers with GPUs. For example, MobileNet, InceptionResNetV2, and InceptionV3 models [31] are trained on the ImageNet database for image recognition. The ImageNet database [32] from Google consists of 14 million images of different objects. There are several pretraining models and databases for image recognition. To use transfer learning, fine-tuning should be applied according to the following steps. First, one should select a model similar to his/her problem. Second, one should decide how many classes one intends to have as output. In this dataset, the problem needed only two classes (ASD and TD) as shown in Figure 3. Third, the network architecture of the model is used as a fixed feature extractor for the dataset. After that, one should initialize all the weights randomly and train the model according to the dataset (in this case ASD and TD). The input image size is 224∗224∗3. The model's custom uses the model's architecture and weight by adding two dense layers on the top. The first layer has 1,024 neurons and the rule activation function. The Kernel regularizer l2 (0.015) is used to reduce the weights (the use bias is false). The dense layer is followed by a dropout layer with (0.4). The second layer for the output prediction uses the Softmax function.

In this study, the output of this model was autism/nonautism. The RMSprop optimizer was used to reduce the model output error during training by adjusting the custom parameters that are added to the top of the model. Various strategies were used to avoid overfitting of the deep learning models, such as batch-normalization and dropout (0.4), but the models' performance did not improve. To conclude, the best option was to use the early stopping strategy to monitor validation loss with ten patients and stop and save the best performance.

## 3. Results

The models were trained on the cloud using the Google Colab environment with python language, which supports the most popular libraries for deep learning, e.g., TensorFlow and Keras. The declaration epochs number was 100 with an 80 batch size. The results of the MobileNet, Xception, and Inception V3 models are presented in Table 1. However, after ten patients, the training stopped on 33 epochs using an early stopping strategy, and the best performance was saved after training with the MobileNet model. The model achieved 95% accuracy on the validation data and 100% on the training data. Figures 9 and 10 plot the model's training accuracy, validation accuracy, training loss, and validation loss. The other two pretraining models (Xception and InceptionV3) were applied to the same dataset, using the same fine-tuning of the layers and optimizer. The accuracy results on the valuation data were 0.94% for Xception and 0.89% for InceptionV3.

### 3.1. Evaluation Metrics

In this study, several metrics were used to evaluate the classifier of the models, including accuracy, sensitivity, and specificity. Sensitivity assesses whether the model correctly identifies images of faces with Autism (“True Positives”). The model accurately identified them as “Autism Positive,” with 0.97% accuracy. Sensitivity was used to measure how often a positive prediction of ASD was correct. Sensitivity was calculated using formula (2).

(2) $$\begin{array}{c} \text{Sensitivity }\frac{\text{True Positives }}{\text{True Positives}+\text{False positives }}. \end{array}$$

Specificity refers to “True Negatives,” which are images of the faces of nonautism children. It measures how often a negative prediction is correct. The model accurately identified them as “Autism Negative,” with 0.93% accuracy. Specificity was calculated using formula (4).

(3) $$\begin{array}{c} \text{specificity}=\frac{\text{True Negatives}}{\text{True Negatives}+\text{False Negatives}}\times 100\%, \end{array}$$

(4) $$\begin{array}{c} \text{Accuracy}=\frac{\text{TP}+\text{TN}}{\text{FP}+\text{FN}+\text{TP}+\text{TN}}\times 100\%. \end{array}$$

### 3.2. Confusion Matrix

For True Positives (TP), the model could correctly predict 131 children as having ASD. For True Negatives (TN), the model could correctly predict 136 children as TD.

For False Positives (FP), the model falsely predicted 9 children as TD, but they had ASD. For False Negatives (FN), the model falsely predicted 4 children as ASD, though they did not have ASD. The confusion matrix details are shown in Figure 11.

### 3.3. Web Application for Autism Detection

Python provides a micro web framework, called Flask, to develop a web application to deploy a deep learning model. In this study, the researchers developed a simple web app for autism facial recognition using HTML, CSS, and JS as the front-end and Flask with the trained model's architecture as the back-end. The application supports an easy interactive user interface that enables specialists to test the child's behavioral state through facial features.

Figure 12 shows the home page of the app where the user can click on the “choose file” button, select the folder in which an image of the face is stored, and select the facial image of the child for testing. Then, the image will be uploaded, and the user can click the submit button. The app will test the image using the trained models, and the prediction will appear, as shown in Figure 13.

## 4. Discussion

Diagnosing autism is a complex task because it involves the behavior of humans. Some cases of autism are misdiagnosed in real-life because of the similarities between ASD and other disorders [32]. To develop an application that recognizes autism using facial feature patterns, one needs to collect data from two groups of children, ASD and TD, label the data as the autism group and the nonautism group, and apply deep learning algorithms. To train a deep learning model, the dataset has to be large enough, and the data collection must follow certain standards because only good data will give good results. This study tried various pretraining models and fine-tuned them, including changing the parameters and learning rate, increasing the hidden layer, and adding batch normalization data augmentation. All these techniques were applied to improve the model's performance.  Table 2 summarizes the results of the proposed system compared to the existing system.

A literature review, which was performed to find the best accuracy for this dataset [32], found three studies that used it. The first study was conducted by Mikian Musser [35], who tried to classify ASD and TD using the VGGFace model, achieved 85% accuracy on the validation data. The second study, which was done by Tamilarasi [36] using the MobileNet model, achieved 94% accuracy on the validation data. The third study, which was done by Beary et al. [28], used the VGG19 model to detect autism facial images. They all used the same dataset [32] and achieved at least 0.84% validation accuracy. A fourth study that was done by Jahanara [37], which implemented the ResNet50 pretraining model on a small dataset consisting of faces of 19 TD and 20 ASD children, achieved 89.2% accuracy. The previous studies relied on the classification method without developing an application that facilitates the diagnostic process in a real-world environment through the use of a user interface.

In this study, the researchers experimentally tested three pretraining models (MobileNet, Xception, and InceptionV3) on a dataset [34] and applied the same fine-tuning of the layers and optimizer.  Table 1 shows the results of the models. MobileNet achieved the highest accuracy (95%) on valuation data with 0.97% sensitivity. Xception achieved the highest specificity (0.95%), but the accuracy was 0.94%. InceptionV3 achieved 0.89% accuracy, 0.95% sensitivity, and 0.83% specificity.

However, the classification results of the MobileNet model are promising, and we are in the process of developing an application of it for autism detection using facial features. The web application for autism detection requires the image to be cropped to show only the face for testing. If the facial image has noise or low resolution and consists of a background, which can lead to misclassification. The limitation of using an online dataset can lead to relative deficiencies in which some faces look nonautistic, the quality of some images is low, and the age range is not appropriate. Moreover, there was no other public dataset available on which to validate this methodology and application.

## 5. Conclusions

This study developed a deep learning-based web application for detecting autism using a convolutional neural network with transfer learning. The CNN architecture has appropriate models to extract the features of facial images by creating patterns of facial features and assessing the distance between facial landmarks, which can classify faces into autistic and nonautistic. The researchers applied three pretraining models (MobileNet, Xception, and InceptionV3) to the dataset and used the same fine-tuning of the layers and optimizer to achieve highly accurate results. MobileNet achieved the highest accuracy with 95% on data valuation and 0.97% sensitivity. Xception achieved the highest specificity (0.95%), but the accuracy was 0.94%. InceptionV3 achieved 0.89% accuracy, 0.95% sensitivity, and 0.83% specificity. Therefore, a MobileNet model was used to develop a web app that can detect autism using facial images. Future work will improve this model by increasing the size of the samples and the collected dataset from psychologists' diagnoses of autistic children who vary in age. This type of application will help parents and psychologists diagnose ASD in children. Getting the right diagnosis of autism could help improve the skills of autistic children by choosing a good plan of treatment.

## Figures and Tables

**Figure 1:** The differences in facial features between children with autism in the first row and children without autism in the second row.

**Figure 2:** Autism detection techniques.

**Figure 3:** The architecture of the proposed application.

**Figure 4:** Bar chart showing the number of pictures used to detect autism from the facial image dataset.

**Figure 5:** The architecture of the proposed model (this image is from Zeyad A.T. Ahmed).

**Figure 6:** Convolutional layer with Max-pooling.

**Figure 7:** Convolutional layer with Max-pooling.

**Figure 8:** Node with activation function.

**Figure 9:** Model accuracy.

**Figure 10:** Model loss.

**Figure 11:** Confusion matrix.

**Figure 12:** The home page of the autism web app.

**Figure 13:** The autism detection web page.

**Table 1:** The results of the tested models.

Model	Accuracy	Sensitivity	Specificity
MobileNet	0.95	0.97	0.93
Xception	0.94	0.92	0.95
InceptionV3	0.89	0.95	0.83

**Table 2:** Comparison of the results of the proposed system against existing models.

No.	Author	Year	Dataset	Method	Accuracy	Application deployment
1	Musser [35]	2020	Detect autism from a facial image [32]	VGGFace model	85%	No
2	Beary [28]	2020	Detect autism from a facial image [32]	MobileNet	94%	No
3	Tamilarasi [36]	2020	The dataset included 19 TD and 20 ASD children	ResNet50	89.2%	No
4	Jahanara [37]	2021	Detect autism from a facial image [32]	VGG19	0.84%	No
5	Our proposed model	2021	Detect autism from a facial image [32]	MobileNet	95%	Yes

## Data Availability

This paper uses a publicly available dataset from Kaggle at https://www.kaggle.com/gpiosenka/autistic-children-data-set-traintestvalidate. This dataset consists of 3,014 face images: 1,507 autistic and 1,507 of nonautistic children. The autistic children face images are collected from online sources related to autism disorder, and the nonautistic children face images are randomly collected from the Internet.
